The article "HPV Vaccination Prevalence among Lebanese Female University Students: A Cross-Sectional Study" was published in 2023. Journal: J Environ Public Health.

# HPV Vaccination Prevalence among Lebanese Female University Students: A Cross-Sectional Study

**DOI:** 10.1155/2023/3706466

**Published:** 2023-06-05

**Authors:** Joey El Khoury, Rami Halabi, Mira Hleyhel, Wafaa El Rahman Kishly, Raghid El Khoury, Nadine Saleh

**Affiliations:** ^1^Notre Dame des Secours University Hospital Center, Street 93, Byblos Postal Code 3, Lebanon; ^2^Department of Urology, School of Medicine and Medical Sciences, Holy Spirit University of Kaslik, P.O. Box 446, Jounieh, Lebanon; ^3^Faculty of Public Health, Lebanese University, Fanar, Lebanon

## Abstract

**Background:**

Cervical cancer is the fourth most common cancer in women, worldwide. Most often, cervical cancer is caused by a human papillomavirus (HPV) infection. A lack of studies concerning HPV knowledge and vaccination among the Lebanese population is noticed. We aim to assess the prevalence of HPV vaccine administration among female university students in Lebanon alongside determining the predictors influencing vaccine uptake. Lastly, knowledge scores concerning HPV and HPV vaccination are also computed.

**Methods:**

This is a cross-sectional analytical study. It is an anonymous, online-based, close-ended questions survey conducted between the 24th of February 2021 and the 30th of March 2021. Our questionnaire was addressed to females aged between 17 and 30 years and enrolled in a Lebanese university. The collected data were analyzed using Statistical Package for Social Sciences (SPSS) v.26. We used bivariate analysis to compare the rate of vaccination with different variables. We used the chi-square test for categorical variables and Student's *t*-test for continuous variables. Logistic linear regression was conducted between the state of vaccination and other statistically significant variables from the bivariate analysis.

**Results:**

We have received a total of 454 questionnaires. Among the respondents, only 18.9% had received a minimum of one dose of the HPV vaccine. The mean age of up taking the first dose of the vaccine was 17.5 years. In addition, 48% of the respondents were not willing to take the HPV vaccine during the upcoming year. Barriers to not taking the HPV vaccine were mainly the low levels of knowledge concerning HPV and its vaccine. In the multivariate analysis, three predictors were found to affect the rate of HPV vaccination: university type, paternal educational level, and HPV vaccine knowledge score. In detail, a student enrolled in a public university had 77% likelihood of not being vaccinated. Furthermore, female students with a paternal educational level higher than a university degree had 88% probability of being vaccinated. Finally, every increase in the HPV vaccination knowledge of one point increased the likelihood of being vaccinated by 37%.

**Conclusion:**

A low vaccination rate among female university students in Lebanon was noticed in our study. In addition, a lack of HPV and HPV vaccine knowledge was found in our population. An awareness campaign alongside public vaccination programs is recommended in order to accomplish higher rates of HPV immunization.

## 1. Background

Human papillomaviruses (HPVs) are the predominant etiologies of sexually transmitted diseases. It is estimated that close to 80% of people worldwide would have contracted at least one strain of HPV by the age of 45 [1] and that the estimated global HPV prevalence is 11.7% across all countries. Studies on different Arab nations revealed an HPV infection prevalence of 10.2% and an overall prevalence of 3.7% for high-risk oncogenic HPV types [2]. More than 20 HPV types fall into that category, especially HPV 16 and 18, which are incriminated in the occurrence of cervical cancer. HPV types 6, 11, 42, and 43 fall into the low-risk category [3]. Sexual behavior was identified as the main risk factor for HPV acquisition [4].

Alongside sexual hygiene, preventive measures can be taken to reduce HPV infectivity and transmission. The World Health Organization (WHO) clearly endorses HPV vaccines and encourages nationwide vaccination campaigns, as these vaccines contribute to low mortality rates attributable to cervical cancer. By 2017, according to the WHO worldwide HPV vaccination report, 71 countries (37% of all nations) introduced HPV vaccines in their national immunization schedule for girls, among them only 11 countries (6% of all nations only) also included vaccines for boys [5]. To date, Lebanon lacks a national strategy for mass HPV vaccination, which is unfortunately not mentioned in vaccination calendars.

Since 2006, three vaccines were licensed and put on the market for public use. The first to be licensed is the quadrivalent vaccine or Gardasil, targeting HPV types 6, 11, 16, and 18. The licensure of Gardasil was subsequently followed by the bivalent Cervarix in 2007 directed solely against high-risk types 16 and 18. A more inclusive Gardasil 9 was licensed in 2014, targeting the same strains as Gardasil, in addition to less prevalent types, HPV-31, 33, 45, 52, and finally 58.

In 2016, researchers investigated the evolution of sexual life in Lebanese youth across 17 universities. They found that 15% of surveyed subjects had already engaged in sexual activity and that 20% were regularly sexually active, while only 36% used condoms. This particular risky behavior shows that turning a blind eye toward HPV and the importance of prophylaxis is no longer an option [6].

Local studies set the prevalence of HPV vaccination in female Lebanese school children at 2.5% and 16.5% in a small sample of 215 students of a prestigious private school in Beirut [7, 8]. Unfortunately, a severe lack of literature on the subject exists, since the available studies only concerned a specific population, making any generalization on the subject biased.

Unfortunately, both official national recommendations for cervical cancer screening practices and a national HPV immunization program do not exist in Lebanon [9]. With sexually transmitted disease rates on the rise due to risky behavior among university students [6], specifically HPV, and given the lack of a clear national vision for combatting cervical cancer through vaccination, this study aimed to estimate the prevalence of HPV vaccine uptake in female university students in Lebanon. In addition, we aimed to highlight the determinants of HPV vaccine uptake decision in an effort to ultimately launch the appropriate campaigns.

## 2. Methods

### 2.1. Study Design

This study was an observational cross-sectional study conducted between the 24th of February 2021 and the 30th of March 2021 using the online questionnaire platform, Microsoft Forms.

### 2.2. Ethical Consideration

The study was reviewed and approved by the ethical review board of INSPECT (IRB Approval No. 2022REC-005-INSPECT-01-21). Data were collected anonymously with no identifying or sensitive information. Students were introduced to the subject and the aim of our study. Moving forward in the online questionnaire was considered to be informed consent.

### 2.3. Study Population and Sampling

We included in this study female university students aged between 17 and 30 years and residing in Lebanon. Due to the pandemic and the unreachable target population, we were obliged to resort to a nonprobability sampling method, which is “snowball” sampling, following a “cascading progression.” A network of informants (trustworthy university students) in all the governorates was recruited to aid our sampling efforts and spread our survey to their peers. Our questionnaire was distributed via a URL in addition to an informative text illuminating the aim of our study. This URL was sent via messages to potential respondents and class representatives.

### 2.4. Minimal Sample Size Calculation

Considering that 119638 female students were enrolled in Lebanese universities [10] and that the expected prevalence of HPV vaccination in Lebanon is around 16.5% [7], a minimal sample size of 211 was calculated using the Epi Info™ software v7.2 (confidence level of 95% and an acceptable margin of error of 5%).

### 2.5. Questionnaire

A well-structured questionnaire was developed after a rigorous literature review related to the following research objective: expert opinions on the importance, intelligibility, and clarity of the questionnaire's content were considered before the final version was distributed. An initial stage of preliminary testing took place before surveying to make sure that the phrasing of the questions is clear and to check the length of time till completion of the questionnaire. On average, the questionnaire took 7 minutes to complete.

The questionnaire was divided into 8 sections and a total of 79 questions. The initial four sections collected data related to the sociodemographic and behavioral characteristics as well as the medical history and sexual behavior of the participants. The remaining sections of the survey included questions on attitudes towards HPV vaccination, in addition to questions evaluating participants' knowledge concerning HPV and its vaccine.

### 2.6. Statistical Analysis

The collected data were assembled, coded, and analyzed using SPSS v.26 (IBM SPSS Inc., Chicago, IL, USA). Continuous variables were reported as means and standard deviations (SD), while categorical variables were summarized as frequencies and percentages. Two indexes on the knowledge of HPV and the HPV vaccine were calculated. Every correct answer to single response questions was given 1 point. However, for multiple response questions, every correct answer was given 1 point while not choosing incorrect responses was also rewarded a point. HPV knowledge index was over 28 and the HPV vaccine knowledge index was over 12. In the bivariate analysis, the chi-square test was used for categorical independent variables and an independent sample *T*-test and Fisher's exact test for continuous variables. Finally, a binary logistic regression was used with having been vaccinated with at least one HPV vaccine dose as the dependent variable of interest. We included in the model all the independent variables with a *p* value <0.2 in the bivariate analysis. A *p* value of ≤0.05 as a significant statistical difference and a confidence interval of 95% were considered.

## 3. Results

### 3.1. Sociodemographic, Medical, Behavioral, and Sexual Characteristics

A total of 454 questionnaires were filled by participants who met the inclusion criteria. The age range varied between 17 years and 30 years with a mean of 22.7 years of age (±3.33). The majority (95.2%) of participants were Lebanese and almost half of them were majoring in nonmedical fields. Less than half of the students (39.4%) were enrolled in the Lebanese university (public). Almost half of the participants (44.7%) had a maternal educational level below a university degree and 58.6% had a paternal educational level below a university degree. Concerning previous medical history, only 1.3% had a personal history of cancer and only 1.5% had a familial history of cancer(s) related to HPV. The majority of the participants (94.3%) have never had a sexually transmitted disease. Regarding behavioral characteristics, around half of the students consume alcohol occasionally and 78.9% do not smoke. Concerning sexual behavior characteristics, almost two-thirds of the responders (65.9%) were not sexually active. In addition, only 10% of the currently sexually active participants never used a condom during sexual intercourse. Regarding the usual number of partners, only 3.3% had two or more sexual partners. Additional and detailed results about sociodemographic characteristics, medical history, and behavioral characteristics are found in Table 1.

### 3.2. HPV Vaccination

The prevalence of taking at least one dose of the HPV vaccine was 18.9%. The mean age of taking the first dose was 17.5 years (±4.89 years). The age of first dose administration ranged between 9 years and 30 years. The main reported reasons for not taking the HPV vaccine were not knowing about HPV (31.2%) and its vaccine (26.6%) and not being sexually active (26.3) (Figure 1). Additional descriptive data concerning the HPV vaccination are available in Table 2. In addition, barriers to not taking the vaccine are represented in Figure 1.

### 3.3. HPV Knowledge

The HPV knowledge index varied from 3 to 25 with a mean score of 13.9 over 28. Detailed participants' responses concerning HPV knowledge are presented in Table 3. Regarding the modes of transmission of HPV, 45.3% of the participants reported sexual intercourse, only 12.8% reported skin-to-skin contact, and 18.6% and 19.5% reported nonpenetrative sex and childbirth, respectively. More than half of the participants (58.4%) reported that HPV can be transmitted even in the asymptomatic phase, 26.4% reported that an HPV infection can lead to cervical cancer, and 35.5% reported that HPV can lead to infertility. The majority of the respondents (78.9%) reported that condom use will reduce the possibility of HPV transmission and know that multiple sexual partners can increase the risk of infection (80.6%). Only 11.7% reported that circumcision prevents HPV infection and transmission. More than half of the respondents (58.6%) reported that HPV infections can be present for many years asymptomatically. Finally, only 5.9% of the participants are aware that an HPV infection cannot be tested in men.

### 3.4. HPV Vaccine Knowledge

HPV vaccine knowledge index had a mean of 4.4 over 12 with a standard deviation of 3.4 and ranged between 0 and 12. Detailed respondents' answers to HPV vaccine knowledge questions are presented in Table 4. Around a third of the respondents (33.9%) reported that the youngest age for HPV vaccine administration is 9 years. Only 27.1% reported that HPV vaccination can prevent oropharyngeal cancer, 33.9% reported that it can prevent penile cancer, and 33.3% reported that it can prevent anal cancer. In addition, only 16.5% reported that the HPV vaccine cannot prevent prostate cancer. Less than half (45.4%) reported that HPV vaccination is more effective if given before the first sexual intercourse. Only 28% reported that HPV-vaccinated persons are not fully immunized against HPV infection. Finally, around two-thirds (67.4%) reported that despite a full course of HPV vaccination, it is not safe to have unprotected sex.

### 3.5. Bivariate Analysis

Tables 5–7 showcase the bivariate analysis and different associations between HPV vaccination status and sociodemographic characteristics, medical history and habits (Table 5), sexual behavior (Table 6), and knowledge scores (Table 7).

### 3.6. Multivariate Analysis

Logistic binary regression was performed using the vaccination status variable as the dependent variable. Given that the smallest group of this variable was the HPV-vaccinated group with *N* = 86, we chose the maximal number of predictors (10%) as 8. From the previously performed bivariate analysis, we had a total of eleven variables with a *p* value of less than 0.2. Therefore, the predictors of our multivariate analysis were chosen depending on their relevance and correlation with our dependent variable.  Table 8 shows the final variables that were entered into the model using the forward likelihood ratio (LR) method.

Table 8 also shows the factors associated with having been vaccinated with at least one HPV vaccine dose. Receiving at least one dose of the HPV vaccine was found associated with being enrolled in a private university compared to enrollment in a public university (ORa = 0.228, *p* < 0.001). Higher paternal educational level was significantly associated with having been vaccinated (ORa = 1.881, *p*=0.027). Finally, a higher HPV vaccine knowledge index was significantly associated with being vaccinated where an increase of 1 point in the index was related to a 37% increase in the odds of having been vaccinated with at least one HPV vaccine dose.

## 4. Discussion

Our study explored the prevalence of HPV vaccine administration and associated predictors among 454 Lebanese female university students aged between 17 and 30 years. On the margin, we aimed to calculate knowledge scores of HPV and HPV vaccines to draw the appropriate assumptions.

According to our results, 18.9% of our target population have received at least one vaccination dose by the time of the survey whilst around 13.9% have received the full regimen of 3 consecutive doses. We opted to consider that 18.9% is the prevalence of HPV vaccination among the surveyed, even though the vaccinated might not have reached optimal immunization status. That was decided given that no clear vaccination program was put in motion by the Lebanese state and that the number of doses needed to be considered fully vaccinated is undefined, varying between 2 and 3. A thorough literature search revealed concerning lack of papers on that matter. The only other significant paper of a study among Lebanese female students at the American University of Beirut found that 16.5% of their sample had received the HPV vaccine [7]. However, compared to a younger target population, such as Lebanese female school girls of private schools in Beirut, with an HPV vaccination prevalence of 2.5%, the age gap becomes more apparent. We could assume that, in general, Lebanese females tend to get vaccinated later in life [8]. In fact, we found that the mean vaccination age was 17.5 (±4.89) with an age range between 9 and 30 years. Merely 15.3% of subjects received their first vaccination dose at age 12 or earlier, conforming to the guidelines stated by the Advisory Committee on Immunization Practices in the United States. Another published paper on HPV vaccination rates in neighboring countries of the Middle East (Jordan, Iraq, UAE, and Qatar) found that only 3% of their female citizens had received all vaccine doses and achieved full immunization. The authors explained this low rate by emphasizing the lack of knowledge of cervical cancer and HPV vaccination by their surveyed subjects. When the unvaccinated were asked about their will to take the HPV vaccine in the upcoming year, only 33% showed willingness to be vaccinated. This result is lower compared to neighboring countries where 43.2% were willing to receive the vaccine [11]. In contrast to a developed and liberal nation, such as the United States of America, the Center for Diseases Control and Prevention (CDC) declared that, in 2020, 77.1% of adolescents aged between 13 and 17 were vaccinated against HPV with at least one dose of whom 61.4% were fully vaccinated [12]. The difference in the vaccination rate between the United States of America and our population may be attributable to the difference in economic status, HPV and HPV vaccine knowledge, and awareness campaigns.

The ideal time for HPV vaccination should be before an individual's first sexual relationship [13]. In our study, among all participants with a positive history of sexual activity, we found that 5.5% had already taken the HPV vaccination before their first sexual intercourse and that the mean age of vaccination was 19.6 years old for taking at least one HPV vaccine dose. This constitutes a public health issue since, as stated earlier, HPV is associated with multiple malignant diseases, most notably cervical cancer among others [14]. To concur, Lei et al. calculated an 88% decreased risk of cervical cancer in participants who initiated HPV vaccination before the age of 17 compared to those who had never been vaccinated [15]. Concerning vaccination barriers, we have found that 24.7% have stated that they did not get vaccinated since the idea was never recommended by their primary physician in the first place. Being rarely covered by Lebanese health care providers, 13.4% did not take the vaccine because of its' expensive price on the market. Abi Jaoude et al. stated that 64% of the 228 primary physicians surveyed in the Greater Beirut area considered the price to be the main barrier against HPV vaccination. In addition, the authors concluded that a refund of vaccine costs by healthcare providers can significantly improve vaccination rates [5]. Drawing conclusions from the Australian experience, HPV vaccination rates increased to an astonishing 70% for girls aged between 12 and 13 after reforming their vaccination program and administering all vaccines free of charge [16].

In an effort to better understand the Lebanese vaccination rates, two knowledge scores were computed, an HPV and its vaccination score. We have found that our sample has a mean HPV knowledge score of 13.9 over 28 points (49.64%). Although some of the questions asked may differ, this score can be compared to the 2015 study by Dany et al. that found a mean knowledge score of 52.7%, where scores were calculated for 512 female students attending one of Beirut's universities. These scores reflect female university students' poor-to-moderate knowledge of HPV [7]. In detail, concerning HPV transmission modes, only 12.8% of our responders chose skin-to-skin transmission; however, it is the main transmission route. The majority of our participants knew that condom use during sexual intercourse will only decrease the risk of HPV transmission and will not prevent the risk completely. These results are compatible with the information found in the literature [17]. In addition, only 29.5% knew that smoking can increase the risk of HPV transmission. In their study, Schabath et al. proved that smoking will increase the risk of HPV transmission with an OR of 1.19. They also found that this association is only valid for carcinogenic HPV [18]. Concerning the rate of HPV transmission in circumcised patients, 11.7% knew that circumcision can lower HPV transmission rates. In a trial by Yuan et al., comparing HPV transmission between uncircumcised and circumcised participants, a 35% reduction in the risk of HPV transmission was noticed in the latter category. In addition, HPV is known to lead to infertility. In our study, 35.5% answered positively to this question. HPV infections were found to be potential risk factors for infertility. HPV is to be screened and treated in couples with fertility issues [19] As per the CDC, there is currently no approved test for HPV testing in men contrary to females where HPV can be tested, and a PAP smear can lead to diagnosing cervical cancer [20].

Regarding HPV vaccination knowledge scores, our sample scored an average of 4.4 over 12 (36.6%) allowing us to draw the same conclusion as Dany et al. A severe lack of knowledge about HPV and its vaccine exists among the surveyed, and this issue should be addressed [7].

It is known that HPV vaccination can be given to the patients 9 years of age and older. Less than half of our participants knew that information. In addition, concerning the prevention of HPV-related cancers, the results were underwhelming. The results of the HPV vaccine knowledge score are even lower than the HPV knowledge score and this is related to a lack of education on sexually transmitted diseases in general and HPV in particular.

In our final analysis, the logistic multivariate analysis, we found that being in a private university was a predictor of being vaccinated. This result, as we have already mentioned, is confirmed by the literature and may be related to the financial status of the participants. However, no previously published studies have found the university type to be a predictor of HPV vaccination. In addition, paternal educational level was also found to be a predictor of HPV vaccination. In detail, women with a paternal university degree or higher had an increased probability of being vaccinated. A recent study conducted in Ethiopia has found similar results concerning HPV vaccination and parental educational level [21]. However, we have found a contradictory result in the literature, where Ganczak et al. mentioned in their study conducted in Poland that there is no significant variance in the HPV knowledge between parents from different educational levels [22]. Another contradictory result was noticed in Feiring et al.'s paper published in 2015. In their study, they found that a higher paternal educational level was associated with a decrease in the probability of receiving HPV vaccines. They have also found a significant association between maternal educational level and HPV vaccination likelihood. Additionally, a study conducted in Texas in 2013 has shown that vaccine refusal was more frequent among parents who are more educated [23]. These findings may be explained by the fear of vaccination side effects. Also, the HPV vaccine knowledge score was found to be a predictor of girls' HPV vaccination. These results are in agreement with a published study from Nigeria where an OR of 7.98 was found concerning the rate of HPV vaccination [24]. In our study, being in a medical or nonmedical major was not found to be a predictor of HPV vaccination status contrary to the results found by Dany et al. [7]. Also, HPV vaccination status increased with increasing age [25]. We did not find age to be a significant predictor of HPV vaccination in our study.

Our study allows the collection of large amounts of data via a single survey. This type of survey is cost-effective and time-effective and of high-yield. Concerning weaknesses, our study has some limitations. In our questionnaire, there were little to no open-ended questions and it did not deepen our understanding of the situation, except through prewritten questions. It is considered inflexible. Furthermore, the majority of the questions in our questionnaire targeted a taboo subject. This may induce a response bias, or it may lead to a decrease in the response rate due to the discontinuation of the questionnaire. Also, the response rate cannot be calculated due to the impossibility of knowing the number of people reached. Finally, a selection bias might be present due to the use of a “snowball” method of sampling. We were limited by the online distribution of the questionnaire due to the COVID-19 pandemic. This step may have limited face-to-face questionnaire filling and the ability to clarify litigious questions.

## 5. Conclusion

In summary, HPV and its related diseases, most notably cervical cancer, are an important public health issue that is often overlooked. Passing on to the literature review, we have found an alarming lack of scientific papers discussing HPV and its vaccine in the Lebanese population. Being part of the HPV vaccination primary target population, we surveyed 454 women enrolled in multiple Lebanese universities and aged between 17 and 30 years. To better understand the burden of HPV on Lebanese society, HPV vaccination prevalence was calculated (18.9%) and was considered low. This prevalence can be partly explained by the computed average low-to-moderate HPV vaccination knowledge score of our sample. In addition, and through our multivariate analysis, we found that having a father with a university degree and being enrolled in a private institution both increase the subject's odds of being vaccinated. We could argue that both of these predictors are associated with better economic status, given that the vaccine is expensive and usually not reimbursed by healthcare providers. To date, no national strategy for HPV vaccination has been put in place. If we were to propose a solution to decrease HPV-related morbidity and mortality in the Lebanese population, we would suggest state-sponsored vaccination awareness campaigns to increase knowledge scores. Making the vaccine cheap or even free and available in the Lebanese market will undoubtedly boost the vaccination prevalence and is crucial to the well-being of our society.

## Figures and Tables

**Figure 1:** Barriers for HPV vaccination.

**Table 1:** Sociodemographic, behavioral, and sexual characteristics and medical history of study participants (*n* = 454).

Variable		*n* (%)	Mean ± SD	Min	Max
*Sociodemographic characteristics*					
Age (years)			22.7 ± 3.33	17	30
Nationality	Lebanese	432 (95.2)			
	Others^1^	22 (4.8)			
Major	Medical^2^	219 (48.2)			
	Nonmedical	235 (51.8)			
University	Public	179 (39.4)			
	Private	275 (60.6)			
Family status	Married	39 (8.6)			
	Single	278 (61.3)			
	In a relationship/engaged	137 (30.2)			
Residence	Beirut	95 (20.9)			
	Mount Lebanon	277 (61)			
	Others^3^	82 (18.1)			
Religion	Christian	287 (63.2)			
	Muslim/Druze	179 (27.7)			
	Nonreligious	18 (4)			
Maternal educational level	Less than university degree	203 (44.7)			
	University degree or higher	251 (55.3)			
Paternal educational level	Less than university degree	266 (58.6)			
	University degree or higher	188 (41.4)			

*Medical history*					
Personal history of cancer	Yes^4^	6 (1.3)			
	No	448 (98.7)			
Family history of cancer related to HPV^5^	Yes	7 (1.5)			
	No history	447 (98.5)			
History of sexually transmitted disease	At least once	26 (5.7)			
	Never	428 (94.3)			

*Behavioral characteristics*					
Alcohol consumption	No	167 (3)			
	Frequently	88 (19.4)			
	Occasionally	199 (43.8)			
Smoking	Yes	96 (21.1)			
	No	358 (78.9)			

*Sexual characteristics*					
Age on first sexual intercourse (years)			21.08 ± 4.02	14	30
Condom use	Always	38 (8.4)			
	Frequently	35 (7.7)			
	Never	46 (10.1)			
	Not currently sexually active	335 (73.8)			
Number of partners in general	One	140 (30.8)			
	Two or more	15 (3.3)			
	Not sexually active	299 (65.9)			
Partner(s) gender	Man	145 (31.9)			
	Woman	6 (1.3)			
	Both	4 (0.9)			
	No sexual partner	299 (65.9)			
Sexual preference (multiple choice question)	Anal giving or receptor	7 (1.5)			
	Oral giving or receptor	73 (16.1)			
	Vaginal sex	140 (30.8)			
	Not sexually active	299 (65.9)			

SD: standard deviation. LBP: Lebanese pound. ^1^Other nationalities include Palestinian (*n* = 9), Syrian (*n* = 8), Iraqi (*n* = 3), Filipino (*n* = 1), and Brazilian (*n* = 1). ^2^“Medical students” include students of medicine, nursing, and pharmacy. ^3^Aakar, North, Baalbeck-Hermel, Beqaa, South, and Nabatiyeh. ^4^Breast cancer; CML, non-Hodgkin lymphoma; hodgkin lymphoma (x2); and kidney cancer. ^5^Cervical cancer; penile cancer; anal cancer; and oropharyngeal cancer.

**Table 2:** Description of HPV vaccination variables.

Variable		*N* (%)	Mean ± SD	Min	Max
Age of HPV vaccination uptake (1^st^ dose) (years)			17.5 ± 4.89	9	30
Age of HPV vaccination uptake (1^st^ dose) in a participant with history of sexual activity (years)			19.6 ± 5.15	10	30

HPV vaccine uptake (at least 1^st^ dose)	Yes	86 (18.9)			
	No	368 (81.1)			
HPV vaccine uptake (2^nd^ dose)	Yes	82 (18.1)			
	No	4 (0.9)
	Did not take the first dose	368 (81.1)

HPV vaccine uptake (3^rd^ dose)	Yes	63 (13.9)
	No	19 (4.2)
	Did not take any doses	372 (81.9)

HPV vaccination before first sexual intercourse	Yes	25 (16.1)
	No	130 (83.9)

Do you intend to get the HPV vaccine in the next year	Yes	150 (33)
	No	218 (48)
	Already took a dose	86 (18.9)

Have you ever heard about HPV	Yes	318 (70)
	No	136 (30)

Have you ever heard about HPV vaccine	Yes	303 (66.7)
	No	151 (33.3)

SD: standard deviation.

**Table 3:** Responses to questions about HPV knowledge by the study participants.

Variable		*n* (%)	Mean ± SD	Min	Max
HPV transmission (multiple responses accepted)	**Sexual intercourse**	409 (45.3)			
	**Skin-to-skin contact**	116 (12.8)			
	**Nonpenetrative sex**	168 (18.6)			
	**During birth**	176 (19.5)			
	None of the above	34 (3.8)			

Can you transmit HPV if you are asymptomatic?	**Yes**	265 (58.4)			
	No	13 (2.9)			
	Do not know	176 (38.8)			

Can smoking increase the risk of HPV?	**Yes**	134 (29.5)			
	No	33 (7.3)			
	Do not know	287 (63.2)			

HPV can cause (multiple responses accepted)	**Anal cancer**	136 (12.6)			
	**Genital warts**	174 (16.1)			
	**Cervical cancer**	286 (26.4)			
	**Oropharyngeal cancer**	125 (11.5)			
	**Penile cancer**	136 (12.6)			
	Prostate cancer	70 (6.5)			
	Do not know	156 (14.4)			
	None of the above	0 (0)			

Can HPV lead to infertility?	**Yes**	161 (35.5)			
	No	37 (8.1)			
	Do not know	256 (56.4)			

Condom use will reduce the possibility of HPV infection	**Yes**	363 (78.9)			
	No	90 (19.8)			
	Do not know	1 (0.2)			

Condom use will completely prevent HPV infection	Yes	50 (11.0)			
	**No**	403 (88.8)			
	Do not know	1 (0.2)			

Can circumcision prevent HPV infection and transmission?	**Yes**	53 (11.7)			
	No	156 (34.4)			
	Do not know	245 (54.0)			

Multiple sex partners will increase the risk of infection?	**Yes**	366 (80.6)			
	No	2 (0.4)			
	Do not know	86 (18.9)			

Will sexual intercourse at an early age increase the likelihood of HPV?	**Yes**	162 (35.7)			
	No	81 (17.8)			
	Do not know	211 (46.5)			

Will washing intimal area reduce the risk of HPV?	**Yes**	118 (26)			
	No	147 (32.4)			
	Do not know	189 (41.6)			

Is it possible to have asymptomatic HPV infection for many years?	**Yes**	266 (58.6)			
	No	9 (2)			
	Do not know	179 (39.4)			

Is there any cure for HPV infection?	Yes	111 (24.4)			
	**No**	102 (22.5)			
	Do not know	241 (53.1)			

Can HPV be tested in men?	Yes	232 (51.1)			
	**No**	27 (5.9)			
	Do not know	195 (43.0)			

What are the possible screening tests?	**PAP smear and HPV testing**	296 (65.2)			
	PAP smear alone	111 (24.4)			
	HPV testing alone	47 (10.4)			

When should HPV screening begin?	**Between 21 and 29**	257 (56.6)			
	Younger than 21	81 (17.8)			
	Older than 29	116 (25.6)			

SD: standard deviation. The correct answers are in bold.

**Table 4:** Responses to questions about HPV vaccine knowledge by the study participants.

Variable		*N* (%)	Mean ± SD	Min	Max
The vaccine is divided into 3 doses over 6 months	**Yes**	188 (41.4)			
	No	23 (5.1)			
	Do not know	243 (53.5)			

HPV vaccine can be given from the age of 9	**Yes**	154 (33.9)
	No	76 (16.7)
	Do not know	224 (49.3)

HPV vaccine can prevent oropharyngeal cancer	**Yes**	123 (27.1)
	No	55 (12.1)
	Do not know	276 (60.8)

HPV vaccine can prevent penile cancer	**Yes**	154 (57.9)
	No	37 (8.1)
	Do not know	263 (57.9)

HPV vaccine can prevent prostate cancer	Yes	90 (19.8)
	**No**	75 (16.5)
	Do not know	289 (63.7)

HPV vaccine can prevent anal cancer	**Yes**	151 (33.3)
	No	38 (8.4)
	Do not know	265 (58.4)

Is the vaccine more effective if given before first sexual intercourse?	**Yes**	206 (45.4)
	No	58 (12.8)
	Do not know	190 (41.9)

Persons who received all doses are fully immunized against cervical cancer?	Yes	58 (12.8)
	**No**	187 (41.2)
	Do not know	209 (46.0)

Persons who received all doses are fully immunized against HPV?	Yes	124 (27.3)
	**No**	127 (28)
	Do not know	203 (44.7)

Is it safe to have unprotected sex after HPV vaccination?	Yes	26 (5.7)
	**No**	306 (67.4)
	Do not know	122 (26.9)

Are HPV vaccine side effects limited to mild local reaction?	**Yes**	143 (31.5)
	No	41 (9)
	Do not know	270 (59.5)

Can HPV cause permanent health problems?	Yes	41 (9)
	**No**	195 (43)
	Do not know	218 (48)

SD: standard deviation. The correct answers are in bold.

**Table 5:** Associations between HPV vaccine uptake and sociodemographic, medical history and habits.

Variable			Results		*p* value
			Vaccinated	Non-vaccinated	
*Sociodemographic characteristics*					
Age^*∗*^			23.48	22.5	0.016t

Major^*∗*^		Medical specialty	51 (23.3)	168 (76.7)	0.023c
		Non-medical specialty	35 (14.9)	200 (85.1)	

University^*∗*^		Public	10 (5.6)	169 (94.4)	0.00c
		Private	76 (27.6)	199 (72.4)	

Nationality		Lebanese	84 (19.4)	348 (80.6)	0.227c
		Other^1^	2 (9.1)	20 (90.9)	

Family status		Married	46 (16.5)	232 (83.5)	0.242c
		Single/divorced	32 (23.4)	105 (76.6)	
		In a relationship/engaged	8 (20.5)	31 (79.5)	

Residence		Beirut	17 (17.9)	78 (82.1)	0.298c
		Mount-Lebanon	58 (20.9)	219 (79.1)	
		Other^2^	11 (13.4)	71 (86.6)	

Religion^*∗*^		Christian	64 (22.3)	223 (77.7)	0.033c
		Muslim/druze	18 (12.1)	131 (87.9)	
		Non-religious	4 (22.2)	14 (77.8)	

Maternal educational level^*∗*^		Less than university degree	26 (12.8)	177 (87.2)	0.002c
		University degree or higher	60 (23.9)	191 (76.1)	

Paternal educational level^*∗*^		Less than university degree	30 (11.3)	236 (88.7)	0.000c
		University degree or higher	56 (29.8)	132 (70.2)	

Individual monthly income^*∗*^		Less than 5.000.000LBP	67 (17)	328 (83)	0.043c
		More than 5.000.000LBP	19 (32.2)	40 (67.8)	
*Medical history*					

Cancer history	No		86 (19.2)	362 (80.8)	0.233c
	Yes^3^		0	6 (100)	

Family history of cancer related to HPV^4^	Yes		2 (28.6)	5 (71.4)	0.512c
	No history		84 (18.8)	363 (81.2)	

History of STD	At least once		4 (15.4)	22 (84.6)	0.633c
	Never		82 (19.2)	346 (80.8)	
*Habits*					

Alcohol drinking^*∗*^	No		19 (11.4)	148 (88.6)	0.005c
	Frequently		23 (26.1)	65 (73.9)	
	Occasionally		44 (22.1)	155 (77.9)	

Smoking	Yes		13 (13.5)	83 (86.5)	0.128c
	No		73 (20.4)	285 (79.6)	

c: Chi-square test; t: student's *T*-test; ^*∗*^: variables with significant difference; LBP: Lebanese pounds; STD: sexually transmitted diseases. ^1^: Syrian, Palestinian, Iraqi, Filipino, Brazilian. ^2^: Aakar, North, Baalbeck-Hermel, Beqaa, South, Nabatiyeh. ^3^: breast cancer, CML, non-Hodgkin lymphoma, Hodgkin lymphoma (x2), kidney cancer. ^4^: cervical cancer, penile cancer, anal cancer, oropharyngeal cancer.

**Table 6:** Bivariate analysis of sexual behavior questions.

Variable		Results		*p* value
		Vaccinated	Nonvaccinated	
Age on first sexual intercourse		21.7	20.8	0.247t

Sexual activity	Active	35 (22.6)	120 (77.4)	0.154c
	Not active	51 (17.1)	248 (82.9)	

Condom use in relationship	Never	13 (28.3)	33 (71.7)	0.184c
	Always	8 (21.1)	30 (78.9)	
	Frequently	9 (25.7)	26 (74.3)	
	Not currently sexually active	56 (16.7)	279 (83.3)	

Number of partners usually	One	34 (24.3)	106 (75.7)	0.092c
	Two and more	1 (10)	14 (93.3)	
	Not sexually active	51 (17.1)	248 (82.9)	

Partner(s) gender	Man	32 (22.1)	113 (77.9)	0.472c
	Woman	2 (33.3)	3 (75)	
	Both	1 (25)	4 (66.7)	
	Not sexually active	51 (17.1)	248 (82.9)	

Sexual preference	Anal giving or receptor	2 (28.6)	5 (71.4)	0.426c
	Oral giving or receptor	16 (21.9)	57 (78.1)	
	Vaginal sex	32 (22.9)	108 (77.1)	
	Not active	51 (17.1)	248 (82.9)	

c: chi-square test; *t*: Student's *T*-test.

**Table 7:** Bivariate analysis of vaccine uptake and knowledge scores.

Variable	Results		*p* value
	Vaccinated	Nonvaccinated	
HPV knowledge score^*∗*^	16.7	13.1	<0.01t
HPV vaccine knowledge score^*∗*^	7.43	3.25	<0.01t

^*∗*^: variable with a significant difference; *t*: Student's *T*-test.

**Table 8:** Factors associated with HPV vaccine uptake (at least one dose) among study participants.

		Adjusted odds ratio (ORa)	95% CI of ORa		*p* value
			Lower	Upper	
University	Public (ref)	0.228	0.108	0.479	<0.001
	Private				

Paternal educational level	University degree or higher (ref)	1.881	1.073	3.297	0.027
	Less than a university degree				
HPV vaccine knowledge score		1.378	1.260	1.508	<0.001

CI, confidence interval; OR, odds ratio binary logistic regression was used (*n* = 454).

## Data Availability

The datasets used and/or analyzed during the current study are available from the corresponding author on reasonable request.

## Abbreviations

CDC: Centers for Disease Control and Prevention
COVID-19: Coronavirus disease 2019
CI: Confidence interval
HPV: Human papillomavirus
INSPECT: Institut National de Santé Publique, D'Epidemiologie Clinique et de Toxicologie
ORa: Adjusted odds ratio
PAP: Papanicolaou test
SD: Standard deviation
URL: Uniform resource locators.
